The article "Effect of Carrying out Continuous Nursing Based on Mobile Platform on the Life of Children with Leukemia after Discharge from Hospital" was retracted in 2024. Reasons: signs of a paper mill; suspected computer-generated content; unreliable results or conclusions; concerns about the data.

# Effect of Carrying out Continuous Nursing Based on Mobile Platform on the Life of Children with Leukemia after Discharge from Hospital

**DOI:** 10.1155/2022/7300303

**Published:** 2022-10-05

**Authors:** Lidan Xu, Xueling Han, Ling Li

**Affiliations:** ^1^Pediatric Internal Medicine, Hainan General Hospital, Hainan Affiliated Hospital of Hainan Medical University, China; ^2^Pediatric Outpation & Emergency, Hainan General Hospital, Hainan Affiliated Hospital of Hainan Medical University, China

## Abstract

**Objective:**

To analyze the effect of carrying out continuous nursing based on mobile platform on the life of children with leukemia after discharge.

**Methods:**

A total of 104 children diagnosed with leukemia admitted in Pediatric Internal Medicine, Hainan Provincial People's Hospital, from September 2019 to August 2020 were randomly divided into two groups, observation group and control group, with 52 cases in each group. For the control group, routine follow-up was used for continuous nursing after discharge from hospital, and the observation group was treated with continuous nursing based on mobile platform on the basis of routine follow-up nursing after discharge from hospital.

**Results:**

When discharged from hospital, there was no significant difference in SDS and SAS scores between the two groups (*P* > 0.05). After 8 weeks of discharge, SDS and SAS scores in both groups were significantly decreased, and SDS and SAS scores in the observation group were significantly lower than those in the control group, with statistical significance (*P* < 0.05). After 8 weeks of discharge, the cancer-related fatigue score of the observation group was significantly lower than that of the control group, and the difference was statistically significant (*P* < 0.05). When discharged from hospital, there was no significant difference in quality of life between two groups (*P* > 0.05). Eight weeks after discharge, the quality of life in both groups was significantly improved, and the quality of life in the observation group was significantly better than that in the control group; the difference was statistically significant (*P* < 0.05). The occurrence of adverse reactions in the observation group was significantly lower than that in the control group, and the difference was statistically significant (*P* < 0.05).

**Conclusion:**

After children with leukemia were discharged from hospital, medical staff used mobile platform to carry out continuous nursing for them, which could relieve the negative emotions of children, reduce the incidence of adverse reactions, and improve the quality of life. This kind of intervention had promotion value.

## 1. Introduction

Leukemia, commonly known as blood cancer, is mainly caused by the malignant cloning of hematopoietic stem cells in patients with cell apoptosis or the imbalance of differentiation, which belongs to a very serious malignant disease [1]. The World Health Organization's International Agency for Research on Cancer (IARC) produces global estimates for all cancers contained in the GLOBOCAN database, using data from mostly high-quality population-based cancer registries worldwide. An estimated 300,000 new cases of leukemia (2.8% of all new cancer cases) are diagnosed each year globally. It has been estimated that in Western countries, CLL constitutes the most frequent type of leukemia with 25% of cases, CML represents 20% of cases, and AML represents 20% of cases.

At present, in the treatment of children with leukemia, chemotherapy is the main treatment means, but there are many adverse reactions to chemotherapy; the treatment compliance of children is poor, causing serious negative effects on the clinical efficacy of treatment [2, 3]. Under normal circumstances, the children discharged from hospital with leukemia can only be given routine discharge guidance, informing their families of discharge matters needing attention, but cannot effectively improve the resistance to treatment of the children with leukemia, unable to improve the quality of life of the children [4, 5]. In children with ALL, 90% of patients achieve a complete remission, and up to 80% can remain disease free at 5 years following treatment. In adults with ALL, remissions occur in 60% to 80%, while 20% to 35% will maintain a leukemia-free survival. Leukemia is responsible for 2% to 6% of orbital tumors in children. Furthermore, up to 11% of children with proptosis will have some form of acute leukemia.

Modern nursing researchers believe that in the nursing process of children with leukemia, continuity of care is an important part of nursing care, which refers to the continuity of care after the discharge of children with leukemia [6], which involves the hospital, relatives, and the children with leukemia themselves, so that the children still get professional nursing guidance after discharge, can correct the wrong cognition of the knowledge of the disease, promote the recovery of the children, and improve the quality of life of the children [7]. Mobile platform is a common platform for modern people to socialize in recent years. It has the characteristics of real time and convenience, which is in line with the needs of modern continuous care [8]. Learning based on e-learning, being ubiquitous, allows easy access anywhere. The nursing professionals are the most important health workers that use a mobile phone for work. They use their personal mobile phones in order to acquire information and to be in contact with the rest of the health team. Mobile nursing is a platform to spread knowledge about diseases and communicate with patients about complications using mobile apps. The top advantages of using mobile devices by providers as well as patients and how they are transforming healthcare enhance physician efficiency, direct patient management, better point-of-care coordination, etc.

In order to explore the effect of carrying out continuous nursing based on mobile platform on the life of children with leukemia after discharge from hospital, 104 children with leukemia were selected and observed in this study. The report is as follows.

The rest of the article is organized according to the following pattern. Methodology is in Section 2.  Section 3 discusses Results. Discussion is mentioned under Section 4, and the journal is concluded in Section 5.

## 2. Materials and Methods

### 2.1. General Information

A total of 104 children diagnosed with leukemia admitted in Pediatric Internal Medicine, Hainan Provincial People's Hospital, from September 2019 to August 2020 were randomly divided into two groups, observation group and control group, with 52 cases in each group.

The following are the inclusion criteria: individuals meet the diagnostic criteria for children with leukemia that was progressively worsening anemia, early fever, unexplained bleeding, lymph node, and hepatosplenomegaly; expected survival time was greater than 2 years; the individual was in good condition and could accept follow-up work; the children and their families were informed of the study and signed the informed consent.

The following are the exclusion criteria: complicated organic disease or systemic disease; severe dysfunction of liver and kidney function; cognitive impairment or a history of mental illness; and those who voluntarily applied to withdraw from this research.

There was no statistically significant difference in general information between the two groups (*P* > 0.05), which are meant to be comparable. General information is shown in Table 1.

### 2.2. Methods

For the control group, routine follow-up was used for continuous nursing after discharge from hospital, such as health information before transfer, regular follow-up, and daily attention manual distribution.

The observation group was treated with continuous nursing based on mobile platform on the basis of routine follow-up nursing after discharge from hospital: explain to children with leukemia and their families the significance, purpose, and methods of implementing continuous care based on mobile platforms before leaving the hospital; children are required to pay attention to the mobile platform inside the hospital, and the nursing staff would carry out the corresponding operation, regularly pushing knowledge about leukemia, such as the daily lifestyle and healthy diet of leukemia patients; use mobile platform to answer questions and communicate with each other; remind the children to report their condition and medication to the medical staff regularly through the mobile platform; conduct online discussions at 19:00 every night through voice and so on to encourage children to speak actively and exchange experiences and encourage children to understand other people's lifestyles, thereby improving the patient's own nursing ability [9]; answer the questions raised by the children, and remind them to return to the hospital on time; and inform children that they need to maintain good living habits in daily life to avoid a series of adverse reactions in the treatment process. For children with more problems or more serious negative emotions, personalized education and psychological intervention could be carried out through the mobile platform, and voice communication could be conducted when it was necessary to solve the difficulties of children in a timely manner.

### 2.3. Observational Index

The observation indexes included negative emotions, cancer-related fatigue, quality of life, and the occurrence of adverse reactions, as follows:

1. Negative emotions: Self-Rating Anxiety Scale (SAS) is a method of measuring levels of anxiety in patients who have anxiety-related symptoms. The scale focuses on the most common general anxiety disorders; coping with stress typically causes anxiety. Each question is scored on a scale of 1-4 (none or a little of the time, some of the time, good part of the time, most of the time). There are fifteen questions worded toward increasing anxiety levels and five questions worded toward decreasing anxiety levels. The scores range from 20 to 80 [10]. Self-Rating Depression Scale (SDS) is a method for measuring depression level. SDS scores are classified as normal (<50), mild depression (50 to 59), moderate to marked major depression (60 to 69), and severe to extreme major depression (>70). The raw score can be converted to an SDS Index score by multiplying the raw score times 1.25 [11]. SDS was used to evaluate the negative emotions before discharge and 8 weeks after discharge, respectively. The lower the SAS and SDS scores, the more mild the anxiety and depression, and the lesser negative emotions.
2. Cancer-related fatigue: 8 weeks after discharge, patients in both groups were evaluated by the self-rating scale for cancer-induced fatigue [12]; the lower the score, the lesser cancer-related fatigue.
3. Quality of life: the quality of life of the children was assessed using the Cancer Quality of Life Inventory EORTC QLQ-C30 [13]; it stands for European Organization for Research and Treatment of Cancer. The higher the EORTC QLQ-C30 score, the better the patient's quality of life. It is designed to measure cancer patients' physical, psychological, and social functions. The questionnaire is composed of multi-item scales and single items.
4. Occurrence of adverse reactions: the adverse reactions are oral infection, gastrointestinal reaction, perianal infection, hair loss, skin and mucosal bleeding, and hyperuricemia.

### 2.4. Statistical Method

SPSS 20.0 statistical software was used for data analysis, measurement data was expressed as *x* ± *s*, and the comparison of the means between the two groups was adopted by a *t* test. A paired *t* test was used before and after intervention in the same group. Enumeration data were expressed as %, and *χ*^2^ test was used for comparison. *P* < 0.05 was considered statistically significant.

## 3. Results

### 3.1. Contrast Results of Negative Emotions

When discharged from hospital, there was no significant difference in SDS and SAS scores between the two groups (*P* > 0.05). After 8 weeks of discharge, SDS and SAS scores in both groups were significantly decreased, and SDS and SAS scores in the observation group were significantly lower than those in the control group, with statistical significance (*P* < 0.05). Contrast results of negative emotions are shown in Table 2.

### 3.2. Contrast Results of Cancer-Related Fatigue

After 8 weeks of discharge, the cancer-related fatigue score of the observation group was significantly lower than that of the control group, and the difference was statistically significant (*P* < 0.05). Contrast results of cancer-related fatigue are shown in Table 3.

### 3.3. Contrast Results of Quality of Life

When discharged from hospital, there was no significant difference in quality of life between two groups (*P* > 0.05). Eight weeks after discharge, the quality of life in both groups was significantly improved, and the quality of life in the observation group was significantly better than that in the control group; the difference was statistically significant (*P* < 0.05). Contrast results of quality of life are shown in Table 4.

### 3.4. Contrast Results of Occurrence of Adverse Reactions

The occurrence of adverse reactions in observation group was significantly lower than control group, and the difference was statistically significant (*P* < 0.05). Contrast results of occurrence of adverse reactions are shown in Table 5.

## 4. Discussion

Due to the toxic and side effects of drugs, the treatment compliance of children with leukemia is poor, and it is more difficult to strictly follow the medical advice due to the lack of continuous nursing guidance after discharge, which is very unfavorable to improve the treatment effect and prognosis [14, 15]. After children with leukemia are discharged from hospital, the nursing staff will apply the mobile platform to carry out continuous nursing, which can enable the medical staff to closely combine with the patients [16], and children with leukemia lack the knowledge of disease and nursing in their daily care. By using a mobile platform, medical staff can regularly release publicity materials and the contents of the next phase of prognosis, so that children and their families can have a comprehensive understanding of the knowledge of disease and nursing [17, 18]. Continuous nursing intervention can enable patients to receive continuous nursing guidance after they leave the hospital and go home. It can effectively promote patients' rehabilitation, reduce the rate of readmission, and improve the quality of life of patients [19]. Relevant studies have shown that continuous nursing guidance for children with leukemia through mobile platform can stimulate their own potential, fully mobilize their own resources, and improve their self-care ability and coping ability at home after discharge [20, 21].

The results of this study showed that when discharged from hospital, there was no significant difference in SDS and SAS scores between the two groups (*P* > 0.05). After 8 weeks of discharge, SDS and SAS scores in both groups were significantly decreased, and SDS and SAS scores in the observation group were significantly lower than those in the control group, with statistical significance (*P* < 0.05). After 8 weeks of discharge, the cancer-related fatigue score of the observation group was significantly lower than that of the control group, and the difference was statistically significant (*P* < 0.05). When discharged from hospital, there was no significant difference in quality of life between two groups (*P* > 0.05). Eight weeks after discharge, the quality of life in both groups was significantly improved, and the quality of life in the observation group was significantly better than that in the control group, the difference was statistically significant (*P* < 0.05). The occurrence of adverse reactions in observation group was significantly lower than control group, and the difference was statistically significant (*P* < 0.05).

## 5. Conclusion

In conclusion, after children with leukemia were discharged from hospital, medical staff used a mobile platform to carry out continuous nursing for them, which could relieve the negative emotions of children, reduce the incidence of adverse reactions, and improve the quality of life. This kind of intervention had promotion value.

## Figures and Tables

**Table 1:** General information.

General information		Observation group	Control group	*P*
Cases		52	52	>0.05
Gender	Boy	25	28	>0.05
	Girl	27	24	
Age (average)		12.14 ± 3.04	12.09 ± 3.71	>0.05
Types of leukemia	Acute myeloid leukemia	24	27	>0.05
	Chronic myelogenous leukemia	16	14	
	Acute lymphoblastic leukemia	12	11	
Clinical staging	Chronic phase	26	27	>0.05
	Acceleration phase	13	14	
	Acute change phase	13	11	
Risk classification	High risk	11	12	>0.05
	Middle risk	15	17	
	Standard risk	26	23	

**Table 2:** Contrast results of negative emotions.

Groups		Observation group	Control group	*t*	*P*
SDS	On discharge	46.04 ± 2.12	45.91 ± 3.07	1.142	>0.05
	8 weeks after discharge	32.06 ± 3.08	39.52 ± 2.93	11.658	<0.05
SAS	On discharge	55.12 ± 4.52	54.20 ± 3.45	0.604	>0.05
	8 weeks after discharge	38.61 ± 2.33	45.17 ± 3.84	8.521	<0.05

**Table 3:** Contrast results of cancer-related fatigue.

Groups	Observation group	Control group	*t*	*P*
Cognition	3.77 ± 0.41	5.36 ± 0.58	12.188	<0.05
Behavior	4.11 ± 0.62	5.68 ± 0.52	12.631	<0.05
Perception	3.37 ± 0.39	4.45 ± 0.48	10.862	<0.05
Emotion	4.12 ± 0.33	5.42 ± 0.60	9.841	<0.05

**Table 4:** Contrast results of quality of life.

Groups		Observation group	Control group	*t*	*P*
Quality of life	On discharge	45.27 ± 4.08	47.01 ± 3.65	2.951	>0.05
	8 weeks after discharge	72.52 ± 2.96	58.44 ± 3.05	9.375	<0.05

**Table 5:** Contrast results of occurrence of adverse reactions.

Groups	Observation group	Control group	*P*
Oral infection	1 (1.92%)	4 (7.69%)	<0.05
Gastrointestinal reaction	3 (5.77%)	6 (11.54%)	<0.05
Perianal infection	1 (1.92%)	3 (5.77%)	<0.05
Hair loss	2 (3.85%)	5 (9.62%)	<0.05
Skin and mucosal bleeding	0 (0.00%)	3 (5.77%)	<0.05
Hyperuricemia	1 (1.92%)	5 (9.62%)	<0.05
Total incidence	8 (15.38%)	26 (50.00%)	<0.05

## Data Availability

The data used to support the findings of this study are included within the article.
